The article "Coronary CTA to Investigate Predictive Value of Left Atrial Appendage for Cardiogenic Stroke in Patients with Nonvalvular Atrial Fibrillation" was published in 2020. Journal: Biomed Res Int.

# Coronary CTA to Investigate Predictive Value of Left Atrial Appendage for Cardiogenic Stroke in Patients with Nonvalvular Atrial Fibrillation

**DOI:** 10.1155/2020/7351876

**Published:** 2020-10-15

**Authors:** Runrong Wang, Chunhong Hu, Zheng Li, Shuai Zhang, Wei Li, Hongling Hou

**Affiliations:** ^1^Department of Radiology, The First Affiliated Hospital of Soochow University, Suzhou, Jiangsu Province 215006, China; ^2^Department of Radiology, Medical Imaging Center, The Affiliated Hospital of Yangzhou University, Yangzhou, Jiangsu Province 225001, China; ^3^Department of Neurology, The Affiliated Hospital of Yangzhou University, Yangzhou, Jiangsu Province 225001, China; ^4^Department of Cardiology, The Affiliated Hospital of Yangzhou University, Yangzhou, Jiangsu Province 225001, China

## Abstract

**Purpose:**

To investigate the predictive value of changes in LAA size and function for cardiogenic stroke (CS) in patients with NVAF by coronary CTA examination. *Materials and Method*. 179 patients with NVAF were selected and grouped according to the outbreak of acute ischemic stroke and TIA within 2 years after coronary CTA examination. Those who met the criteria for CS were selected as cases (87 patients), and those neither stroke nor TIA as controls (92 patients). LAA size of selected patients was measured and data postprocessing was performed. The differences of baseline data and LAA parameters between groups were analyzed. The impacts of BMI, hyperlipidemia, the duration of AF, the LAAOA Index, and the LAAEF on CS were assessed by binary logistic regression. The predictive abilities of LAAOA Index, LAAEF, and the combined predictor were assessed by ROC curves.

**Results:**

Proportions of BMI ≥ 25, prevalence of hyperlipidemia, duration of AF, and LAAODmax, LAAODmin, LAAOA, LAAVmax, and LAAVmin with their correction index were greater in cases than controls. The LAAEF was lower in cases than that in controls. The binary logistic regression model showed an increase in LAAOA Index (*P* = 0.005) and a decrease in LAAEF (*P* < 0.001) were independent risk factors for CS. ROC curve analysis showed that the optimal cutoff values of LAAOA Index and LAAEF to predict CS were 3.16 cm^2^/m^2^ and 38.71%, with AUC value of 0.712 and 0.734, respectively. The LAAOA Index-LAAEF combined predictor (AUC value = 0.786) was likely superior to either LAAOA Index or LAAEF.

**Conclusions:**

Coronary CTA can provide additional valuable parameters, as a by-product of coronary artery assessment without additional radiation dose, for the risk assessment of CS in patients with NVAF. Coronary CTA may make up for the limitation of single indicator of CHA_2_DS_2_-VASc in guiding anticoagulation program, to reduce the incidence of embolism and bleeding events.

The article "Coronary CTA to Investigate Predictive Value of Left Atrial Appendage for Cardiogenic Stroke in Patients with Nonvalvular Atrial Fibrillation" was published in 2020. Journal: Biomed Res Int.

## 1. Introduction

As defined in the 2014 AHA/ACC/HRS guideline for the management of patients with atrial fibrillation, nonvalvular atrial fibrillation (NVAF) refers to an atrial fibrillation that occurs in patients without rheumatic mitral valve disease, mechanical or biological valve replacement, and mitral annuloplasty [1]. With the aging of the population structure, the incidence of NVAF has increased year by year. According to a recent epidemiological survey, the incidence of NVAF is about 10% in people over 75 years old [2, 3]. The annual incidence of cardiogenic stroke in patients with NVAF is about 5%, which is 2 to 7 times that of sinus rhythm [4]. Compared with other types of ischemic stroke, cardiogenic stroke has higher hemorrhagic transformation, disability, and mortality and the prognosis is poor [5, 6]. Cardiogenic stroke also has a high rate of early recurrence, with a recurrence rate of approximately 12% within 2 weeks of the onset of initial symptoms [7, 8]. How to effectively control and prevent cardiogenic stroke is a challenge for the academic community, and exploring the risk factors associated with cardiogenic stroke is the essential point. The left atrial appendage (LAA) as the main part of the formation of responsible emboli in cardiogenic stroke in patients with atrial fibrillation, and its influence on the progress of disease has become the focus of current research. Currently, clinicians generally rely on the CHA_2_DS_2_-VASc scoring system to assess the risk of embolism in patients with atrial fibrillation and to guide anticoagulant therapy. However, a single assessment indicator often fails to meet practical needs. The aim of this study was to investigate the effect of quantitative indicators of anatomy and function of LAA on the risk of cardiogenic stroke in patients with NVAF by coronary CTA and to provide valuable imageology reference for the design of clinical anticoagulation program.

## 2. Materials and Methods

### 2.1. Research Object

In the beginning, a total of 385 patients with NVAF who underwent coronary CTA examination to assess the condition of coronary arteries between January 2014 and June 2017 were selected. Atrial fibrillation was diagnosed according to the conventional 12-lead electrocardiogram (ECG) or 24-hour Holter. Collect demographic data, clinical history data, and laboratory and imageology findings of these patients, and exclude the following: (1) history of rheumatic mitral valve disease, congenital heart disease, and cardiomyopathy; (2) history of various types of cardiac surgery; (3) history of pulmonary embolism or deep vein thrombosis; (4) coronary CTA scan range does not include the whole LAA, or LAA is poorly displayed; (5) and presence of LAA thrombosis. Consequently, 326 patients were enrolled and were followed up for 2 years. The patients were classified based on the outbreak of acute ischemic stroke and transient ischemic attack (TIA) within 2 years after coronary CTA examination and were further classified based on the TOAST classification criteria. During the follow-up period, 147 patients were excluded including those who met the TOAST criteria for noncardiogenic stroke, patients with TIA attacks, and some lost to follow-up. Of the remaining 179 cases, 87 patients with cardiogenic stroke were selected as the case group and 92 patients with neither acute ischemic stroke nor TIA during the follow-up period were selected as the control group. The diagnosis of stroke and TIA is based on the results of head MR examination and clinical manifestations and is consensually diagnosed by two neurologists with more than 10 years of practicing experience. Because the age composition of population in this study was mainly elderly (63.9 ± 8.4 yrs), the overall compliance with long-term anticoagulation therapy was poor. In addition, some patients discontinued the drug due to bleeding risk or other factors during the follow-up period. Therefore, the proportion of patients continuously using anticoagulants in both groups in this study was low, and there was no statistical difference between the groups (9.2% *vs* 12.0%, *X*^2^ = 0.359, *P* = 0.549). Warfarin was used for anticoagulation in all patients except for one patient who used Dabigatran etexilate in each of the two groups. The study was approved by the ethics committee, and patients who participated in the study signed an informed consent.

The article "Coronary CTA to Investigate Predictive Value of Left Atrial Appendage for Cardiogenic Stroke in Patients with Nonvalvular Atrial Fibrillation" was published in 2020. Journal: Biomed Res Int.

### 2.2. Examination Method

The patients' heart rates were controlled at 50-75 beats/min, and those with a faster heart rate were given oral 25 mg metoprolol. Before the examination, the patients were given breath-holding training. The patients were placed in a supine position in the examination and were scanned at the end of the expiration when holding their breath. The breath holding time was about 4 to 6 seconds. The cardiac CTA scan was performed using a 128-slice CT scanner (SOMATOM Definition AS CT, Siemens Medical, Forchheim, Germany). Scanning parameter was as follows: tube voltage 120~140 KV, tube current 180~200 mAs, automatic matching pitch, collimator width 128 × 0.6 mm, FOV 180~210 mm, convolution kernel B35f and B46f, scanning time 4~6 s. Retrospective ECG gating was used. Scan range was from 1 cm above the tracheal bifurcation to 1 cm below the diaphragm face of the heart. The contrast agent concentration monitoring layer was placed at the root of the ascending aorta, and the scan is initiated when the CT value in the ROI exceeds a preset threshold (160 HU). The contrast agent (Ultravist 370 mg/ml, dose 1.0 ml/kg) in combination with physiological saline 70 ml (20 ml before injection of a contrast agent, 50 ml after injection of a contrast agent) was injected through the median elbow vein at a rate of 5.0 ml/s using a double-tube high-pressure syringe.

## 3. Image Postprocessing and Measurement

Postprocessing and measurement were performed jointly by two radiologists who were blinded to clinical data (including history of stroke/TIA), using dedicated software (Syngo MMWP VE32D, Siemens Medical, Forchheim, Germany) on the workstation. Consensus was obtained for each case. In the beginning, with the assistance of a cardiologist, the two radiologists were trained on an initial sample of 20 cases to standardize the image reconstruction of LAA and parameter measurement. The maximum and minimum diameters of the left atrial appendage orifice (LAAODmax and LAAODmin), the left atrial appendage orifice area (LAAOA), the left atrial appendage depth (LAAD), the left atrial appendage volume (LAAV), the correction index of corresponding parameter, and the left atrial appendage emptying fraction (LAAEF) were obtained as follows: (1) the multiplanar reformation (MPR) was performed at the junction of LAA and left atrium (reference demarcation mark: a line connecting 1~2 cm below the left upper pulmonary vein orifice with the left coronary artery originating position), and a short-axis view of the LAA orifice was obtained that can be used to measure the LAAODmax, LAAODmin, and LAAOA (see Figures 1(a)–1(c)); (2) curved planar reformation (CPR) along the LAA long-axis and measuring the distance from the center of the LAA orifice to the LAA vertex on the CPR recombination image to obtain the LAAD (see Figures 1(d)–1(e)); (3) using the reconstructed images of each phase, manually tracing the endocardial border of the individual short-axis segments by the volumetric measurement tool to calculate the LAAV of each phase by the layer-stacking method (see Figure 2), and determining the maximum LAAV (LAAVmax) and the minimum LAAV (LAAVmin); (4) using the body surface area (BSA) to correct each measured parameter to obtain the correction index of the corresponding parameter: value index = value/BSA; and (5) the LAAEF was calculated using the following equation: LAAEF = (LAAVmax − LAAVmin)/LAAVmax × 100%.

### 3.1. Statistical Analysis

Statistical analysis was performed using SPSS 17.0 and Med Calc 15.0 statistical software. Continuous data close to the normal distribution were expressed as mean ± standard deviation ($\bar{x}\pm s$), and nonnormally distributed data were expressed as median (lower quartile − upper quartile). Categorical data were presented as absolute numbers (percentages). Differences in continuous variables between the two groups were assessed using Student's *t*-test or Mann–Whitney *U*-test, as appropriate. Differences in categorical variables between the two groups were assessed using a Pearson chi-square test. The difference was considered statistically significant at *P* < 0.05. The impacts of body mass index (BMI), hyperlipidemia, the duration of atrial fibrillation, LAAOA Index, and LAAEF on cardiogenic stroke were assessed by a binary logistic regression analysis, and the continuous data had been grouped into quartiles. We adopted a forward stepwise regression method based on maximum likelihood estimation for the variable screening method. To assess the ability of LAAOA Index, LAAEF, and the combined predictor of LAAOA Index and LAAEF in predicting cardiogenic stroke, receiver operating characteristic (ROC) curves were constructed. The AUC value (area under the ROC curve) was used as a scalar measure to assess the performance of each parameter. The AUC value for different parameters were compared by a *Z* test; *P* < 0.05 was considered statistically significant.

The article "Coronary CTA to Investigate Predictive Value of Left Atrial Appendage for Cardiogenic Stroke in Patients with Nonvalvular Atrial Fibrillation" was published in 2020. Journal: Biomed Res Int.

## 4. Results

The demographic and clinical data of the two groups are listed in Table 1. The proportion of overweight or obesity (BMI ≥ 25) (71.3% *vs* 51.1%, *X*^2^ = 7.645, *P* = 0.006) and the prevalence of hyperlipidemia (59.8% *vs* 42.4%, *X*^2^ = 5.404, *P* = 0.020) in the case group were higher than those in the control group. The duration of atrial fibrillation was longer in the case group than that in the control group [5 (3-9) yrs *vs* 4 (2-7) yrs, *Z* = −2.995, *P* = 0.003]. There were no significant differences between two groups in terms of gender, age, body surface area (BSA), smoking history, drinking history, hypertension, diabetes, coronary heart disease, CHA_2_DS_2_-VASc score, continuous use of anticoagulants during the follow-up period, and atrial fibrillation type (paroxysmal atrial fibrillation *vs* persistent or permanent atrial fibrillation, similarly hereinafter).

The parameters derived from coronary CTA are shown in Table 2. The LAAODmax (3.31 ± 0.38 cm *vs*2.97 ± 0.38 cm, *t* = 5.862, *P* < 0.001) with its correction index (1.80 ± 0.21 cm/m^2^*vs*1.64 ± 0.24 cm/m^2^, *t* = 4.783, *P* < 0.001), LAAODmin (2.18 ± 0.32 cm *vs*1.93 ± 0.33 cm, *t* = 5.212, *P* < 0.001) with its correction index (1.19 ± 0.17 cm/m^2^*vs*1.06 ± 0.19 cm/m^2^, *t* = 4.647, *P* < 0.001), LAAOA (5.90 ± 1.36 cm^2^*vs*4.80 ± 1.14 cm^2^, *t* = 5.820, *P* < 0.001) with its correction index (3.20 ± 0.71 cm^2^/m^2^*vs*2.65 ± 0.64 cm^2^/m^2^, *t* = 5.481, *P* < 0.001), LAAVmax (14.58 ± 3.73 ml *vs*12.02 ± 3.16 ml, *t* = 4.946, *P* < 0.001) with its correction index (7.91 ± 1.92 ml/m^2^*vs*6.61 ± 1.68 ml/m^2^, *t* = 4.826, *P* < 0.001), and LAAVmin (9.27 ± 2.69 ml *vs*6.66 ± 2.38 ml, *t* = 6.877, *P* < 0.001) with its correction index (5.03 ± 1.40 ml/m^2^*vs*3.67 ± 1.28 ml/m^2^, *t* = 6.823, *P* < 0.001) in the case group were greater than those in the control group. The case group tended to has lower LAAEF (36.20 ± 10.54% *vs*45.25 ± 10.07%, *t* = −5.875, *P* < 0.001) than the control group. There were no statistically significant differences between two groups in the ratio of LAAODmax to LAAODmin (1.53 ± 0.16*vs*1.56 ± 0.21, *t* = −1.280, *P* = 0.202) and the LAAD (4.61 ± 0.56 cm *vs*4.45 ± 0.71 cm, *t* = 1.579, *P* = 0.116) with its correction index (2.51 ± 0.31 cm/m^2^*vs*2.46 ± 0.44 cm/m^2^, *t* = 0.801, *P* = 0.425).

The article "Coronary CTA to Investigate Predictive Value of Left Atrial Appendage for Cardiogenic Stroke in Patients with Nonvalvular Atrial Fibrillation" was published in 2020. Journal: Biomed Res Int.

The variables of LAAOA Index, LAAEF, BMI, hyperlipidemia, and the duration of atrial fibrillation were incorporated into the binary logistic regression model. Among these variables, LAAOA Index (*P* = 0.005) and LAAEF (*P* < 0.001) were statistically significant; the BMI (*P* = 0.205), hyperlipidemia (*P* = 0.222); and the duration of atrial fibrillation (*P* = 0.059) were not statistically significant. The resulting logistic regression model was statistically significant (*X*^2^ = 42.250, *P* < 0.001). After adjusting for the BMI, hyperlipidemia, and the duration of atrial fibrillation, the binary logistic regression model showed that an increase in LAAOA Index and a decrease in LAAEF were independent risk factors for cardiogenic stroke. The cardiogenic stroke risk of the highest quartile of LAAOA Index was 5.826 times (95% CI = 2.167~15.661, *P* < 0.001) the lowest quartile, and the risk of the lowest and the second lowest quartile of LAAEF was 8.255 times (95% CI = 2.929~23.264, *P* < 0.001) and 3.081 times (95% CI = 1.166~8.139, *P* = 0.023) the highest quartile, respectively. The model correctly classified 71.5% of the research objects. The model's sensitivity was 70.1%, its specificity was 72.8%, its positive predictive value was 70.9%, and its negative predictive value was 72.0% (Table 3).

The receiver operating characteristic (ROC) curves of the LAAOA Index, the LAAEF and the combined predictor of LAAOA Index and LAAEF showed that the AUC value of LAAOA Index was 0.712 (95% CI = 0.639-0.777, *Z* = 5.570, *P* < 0.0001), the optimal cutoff value was 3.16 cm^2^/m^2^ with a sensitivity of 54.02% and a specificity of 78.26%; the AUC value of LAAEF was 0.734 (95% CI = 0.663-0.797, *Z* = 6.305, *P* < 0.0001), the optimal cutoff value was 38.71% with a sensitivity of 62.07% and a specificity of 75.00%; the AUC value of the LAAOA Index and LAAEF combined predictor was 0.786 (95% CI = 0.718-0.843, *Z* = 8.533, *P* < 0.0001). The difference of the AUC value between the combined predictor and LAAOA Index (0.074, *Z* = 2.667, *P* = 0.0077) and that between the combined predictor and LAAEF (0.052, *Z* = 2.061, *P* = 0.0393) were statistically significant. The combined predictor was likely superior to either the LAAOA Index or LAAEF for predicting cardiogenic stroke. The difference of the AUC value between LAAOA Index and LAAEF was not statistically significant (0.022, *Z* = 0.448, *P* = 0.6544) (see Figure 3).

The article "Coronary CTA to Investigate Predictive Value of Left Atrial Appendage for Cardiogenic Stroke in Patients with Nonvalvular Atrial Fibrillation" was published in 2020. Journal: Biomed Res Int.

## 5. Discussion

Cardiac stroke is an important complication of atrial fibrillation (AF). The incidence of cardiogenic stroke in patients with AF is 5.6 times higher than that of sinus rhythm [9]. Compared with other types of ischemic stroke, cardiogenic stroke has more severe neurological deficits, more associated diseases, and higher recurrence, disability, and mortality [10–13]. The LAA is the main site of emboli formation in cardiogenic stroke in patients with AF. In patients with valvular atrial fibrillation (VAF), about 60% of cardiac thrombosis is formed in the LAA, and the ratio is greater than 90% in patients with nonvalvular atrial fibrillation (NVAF) [14–16]. The LAA is a remnant of the original left atrium of the embryonic period and resembles an irregular tubular diverticulum. There are significant individual differences in the morphology and size of the LAA in the physiological conditions [17, 18]. Therefore, in this study, body surface area (BSA) was used to correct each measured parameter to reduce the bias caused by this individual differences. The LAA has an active diastolic and contraction function, and it can exert certain adaptive adjustment effect when the volume load of the atrium is abnormal. When the blood flow in the LAA passes by the normal flow state and flow rate, it is difficult to form a thrombus. Pathological conditions such as atrial fibrillation can lead to changes in the structure and function of the LAA, causing eddy currents and stasis in the blood flow, which in turn leads to thrombosis [19, 20]. When the thrombus in the LAA is organized, detached, and ejected through the left ventricle, it will cause distal arterial embolization of the systemic circulation. About 80% of the embolic events occur in the cerebral blood vessels, leading to cardiogenic stroke [21]. Changes in the structure and function of the LAA affect not only the occurrence of stroke but also the progression and prognosis of stroke [22, 23].

The article "Coronary CTA to Investigate Predictive Value of Left Atrial Appendage for Cardiogenic Stroke in Patients with Nonvalvular Atrial Fibrillation" was published in 2020. Journal: Biomed Res Int.

The result of this study showed that patients with cardiogenic stroke tend to have larger LAA orifices and volumes. In agreement with this result, Khurram et al. reported that the maximum diameter of LAA orifice was positively correlated with the occurrence of cardiogenic stroke [24]. Taina et al. found that the LAA volume in patients with cardiogenic stroke was greater than that in the control group [25]. A study by Burrell et al. showed that patients with the LAA volume > 34 ml have a 7 times increased risk of ischemic stroke and embolic events compared with controls [26]. A larger LAA orifice or volume is more likely to cause a slower flow of blood in the LAA, especially at the part of orifice, and more eddy currents. Slow blood flow and eddy currents increase the chances of platelet aggregation and collision, accelerating platelet function activation, and increasing the risk of thrombosis and cardiogenic stroke. Previous studies have shown that with the progression of AF, there is an anatomic LAA remodeling, which is characterized by an increase in the volume of the LAA, an atrophy in the comb muscles, and an intimal elastic fiber tissue hyperplasia. The anatomic LAA remodeling may be one of the causes of the LAA orifice and volume to be larger in pathological conditions [27]. It is still unknown which one is the main cause of the larger LAA orifice and volume with regard to the anatomic LAA remodeling and hemodynamic changes in AF condition [27]. In view of the duration of atrial fibrillation being longer in the case group than the control group [5(3-9) yrs *vs* 4(2-7) yrs, *Z* = −2.995, *P* = 0.003] in this study and the causes of the difference in LAAOA and LAAV between groups, in addition to individual differences, hypertension, mitral regurgitation, and other factors, the role of atrial fibrillation progression in anatomic LAA remodeling should be considered. This study showed that the differences of the ratio of LAAODmax to LAAODmin (1.53 ± 0.16*vs*1.56 ± 0.21, *t* = −1.280, *P* = 0.202) and the LAAD (4.61 ± 0.56 cm *vs*4.45 ± 0.71 cm, *t* = 1.579, *P* = 0.116) with its correction index (2.51 ± 0.31 cm/m^2^*vs*2.46 ± 0.44 cm/m^2^, *t* = 0.801, *P* = 0.425) between groups were not statistically significant, suggesting that the shape of LAA orifice and the LAA depth were not correlated with cardiogenic stroke in patients with NVAF. This conclusion needs further study to confirm.

Ono and colleagues found that the LAAEF ≤ 21% was independently associated with the LAA thrombosis [28]. Similarly, the case group has a lower LAAEF compared with the control group in this study (36.20 ± 10.54% *vs*45.25 ± 10.07%, *t* = −5.875, *P* < 0.001), suggesting that the LAA emptying function in patients with cardiogenic stroke tends to be weaker. The emptying obstacle of LAA leads to blood stasis and increases the risk of thrombosis and cardiogenic stroke in patients with AF. In the early stage of LAA remodeling in patients with AF, there is a myocardial atrophy and necrosis, with inflammatory cell infiltration, then endocardial elastic fiber tissue proliferation, abnormal deposition of collagen, and finally due to limited metalloproteinase activity; the LAA comb muscles are surrounded by collagen and its function is impaired, leading to the LAA emptying dysfunction, manifested by a decreased LAAEF and blood flow rate [28, 29]. The pathological changes of the LAA remodeling in patients with AF are progressively aggravated with the prolongation of the disease course of AF [27]. Due to the longer duration of atrial fibrillation in the case than control group in this study, the lower LAAEF in the case group should be related to the pathological process of the LAA remodeling. The widening of LAA orifice and the enlargement of LAA volume make it difficult for the inward movement of LAA wall to cause sufficient emptying, which causes the blood flow in LAA to become slow and stagnant and eddy currents. Severe eddy current can cause damage to the intima and can further aggravate the abnormality of platelet function, coagulation, and fibrinolysis in patients with AF [30]. These factors together constitute the pathological basis of thrombosis, which may lead to the occurrence of cardiogenic stroke.

The article "Coronary CTA to Investigate Predictive Value of Left Atrial Appendage for Cardiogenic Stroke in Patients with Nonvalvular Atrial Fibrillation" was published in 2020. Journal: Biomed Res Int.

For the secondary prevention of cardiogenic stroke in patients with atrial fibrillation, the assessment tool commonly used in clinical anticoagulant therapy is CHA_2_DS_2_-VASc (congestive heart failure, hypertension, age ≥ 75 (doubled), diabetes, stroke (doubled), vascular disease, age 65-74, and sex category (female)). In this study, the demographic and clinical baseline data related to the CHA_2_DS_2_-VASc score of the two groups were overall similar to each other, and there was no statistical difference in the proportion of patients whose CHA_2_DS_2_-VASc scores ≥ 2 between the two groups (74.7% *vs* 71.7%, *X*^2^ = 0.201, *P* = 0.654). However, a single assessment index often fails to meet the actual needs in clinical practice. For patients with CHA_2_DS_2_-VASc score ≤ 1 or those with ≥2 points with high bleeding risk, the single CHA_2_DS_2_-VASc score can lead to insufficient or excessive anticoagulation, increasing the incidence of embolism and bleeding events [31, 32]. Therefore, it is necessary to explore an assessment tool that is practical, clinically easy to use, and easy to promote for the prophylactic anticoagulant therapy for cardiogenic stroke in patients with atrial fibrillation as a supplement to the CHA_2_DS_2_-VASc score. Transesophageal echocardiography (TEE) can measure the LAA size and assess its function by hemodynamic parameters and can also visually detect the thrombus in LAA. However, as a semi-invasive examination, TEE has limited its clinical application due to its long operation time, low patient compliance, high dependence on the operation technique, potential trauma, and risk of anesthesia. The coronary CTA examination is convenient and noninvasive and has become a routine application of cardiology patients in clinical practice [33–35]. Cardiac computed tomography offers a high spatial resolution and a fast dataset acquisition, and it can provide a detailed characterization of atrial anatomy and has been shown to guide LAA closure or catheter ablation of atrial fibrillation [36]. Lopez-Minguez and colleagues evaluated the measurements obtained using computed tomography (CT), intraoperative transesophageal echocardiography (IOTEE), and angiography to select the size of the closure device in LAA closure. They found that the combination of angiography-CT was the most accurate for the selection of device size [37]. This study shows that coronary CTA can provide a one-stop assessment of the anatomical shape, size, and function of LAA by data postprocessing without additional radiation dose after coronary assessment is completed. We measured the parameters of LAA size and function by coronary CTA and found that an increase in LAAOA Index (*P* = 0.005) and a decrease in LAAEF (*P* < 0.001) are independent risk factors for cardiogenic stroke, and in terms of the ROC curve analysis, the parameters of the LAAOA Index and LAAEF with the AUC value of 0.712 (95% CI = 0.639-0.777, *Z* = 5.570, *P* < 0.0001) and 0.734 (95% CI = 0.663-0.797, *Z* = 6.305, *P* < 0.0001), respectively, have medium predictive value for cardiogenic stroke in patients with NVAF. The LAAOA Index and LAAEF combined predictor with an AUC value of 0.786 (95% CI = 0.718-0.843, *Z* = 8.533, *P* < 0.0001) was superior to either LAAOA Index (*Z* = 2.667, *P* = 0.0077) or LAAEF (*Z* = 2.061, *P* = 0.0393), which indicates that a comprehensive consideration of the two factors likely leads to a more accurate judgment.

The article "Coronary CTA to Investigate Predictive Value of Left Atrial Appendage for Cardiogenic Stroke in Patients with Nonvalvular Atrial Fibrillation" was published in 2020. Journal: Biomed Res Int.

There are several potential limitations to this study. The sample size of two groups was relatively small, thus limiting the power for multivariable analyses. In addition, the predictive values of LAAOA Index and LAAEF were both medium, and neither sensitivity nor specificity of the cutoff values of LAAOA Index (3.16 cm^2^/m^2^, with a sensitivity of 54.02% and a specificity of 78.26%) and LAAEF (38.71%, with a sensitivity of 62.07% and a specificity of 75.00%) was satisfactory. The reason may be that the two groups were both composed of patients with AF, and furthermore, there was no disparity of median duration years of AF between them [5 (3-9) years *vs* 4 (2-7) years, *Z* = −2.995, *P* = 0.003]. Therefore, the results from this study are likely more suitable for the population of AF. To obtain more valuable findings, corresponding patients without AF should be enrolled, and multicenter studies should be conducted in the future. Furthermore, this study lacks the comparison with other imaging techniques. It is expected that cases from transesophageal echocardiography, especially positive cases with LAA thrombi, will be enrolled to reinforce the study results. Finally, some unmeasured confounding may exist owing to the limitation of the retrospective study. Although there was no statistical difference in the proportion of anticoagulants used in the two groups, there were some false negative cases caused by the anticoagulation status. Therefore, the results need to be further verified by prospective studies.

## 6. Conclusions

LAAOA Index and LAAEF have predictive value for cardiogenic stroke in patients with NVAF, and the value of the two parameters combined is likely higher. In addition, the coronary CTA is able to provide additional valuable imageology parameters, as a by-product of coronary artery assessment without additional radiation dose, for the risk assessment of cardiogenic stroke in NVAF, especially those with low risk of CHA_2_DS_2_-VASc score, contraindication, or intolerance to TEE. Moreover, coronary CTA may join in guiding the design of a clinical anticoagulation program to make up for the limitation of a single indicator of CHA_2_DS_2_-VASc score, so as to reduce the probability of insufficient or excessive anticoagulation and to reduce the incidence of embolism and bleeding events.

## Figures and Tables

**Figure 1:** An example of cardiac CTA images illustrating the measurement of the left atrial appendage (LAA): (a) locating the LAA orifice in its long-axis view; (b, c) measurements of the maximum and minimum left atrial appendage orifice diameter (LAAODmax and LAAODmin, respectively) and the left atrial appendage orifice area (LAAOA) in the short-axis view; (d, e) by implementing curved planar reformation (CPR) along the LAA long-axis, a straightened LAA is obtained that can be used to measure the left atrial appendage depth (LAAD).

**Figure 2:** Manually tracing the endocardial border of the individual short-axis segments. The long-axis view of the left atrial appendage results from the stacking of multiple short-axis segments, to calculate the left atrial appendage volume (LAAV).

The article "Coronary CTA to Investigate Predictive Value of Left Atrial Appendage for Cardiogenic Stroke in Patients with Nonvalvular Atrial Fibrillation" was published in 2020. Journal: Biomed Res Int.

**Figure 3:** Receiver operating characteristic (ROC) curves comparing parameters for the prediction of cardiogenic stroke. Curves are shown for LAAOA Index, LAAEF, and the combined predictor of LAAOA Index and LAAEF (LAAOA Index-LAAEF combined).

**Table 1:** Comparison of demographic and clinical data between the two groups.

Characteristics	Total (*n* = 179)	Cases (*n* = 87)	Controls (*n* = 92)	Statistic value	*P* value
Sex, *n* (%)					
Male	102 (57.0)	48 (55.2)	54 (58.7)	0.226^#^	0.634
Female	77 (43.0)	39 (44.8)	38 (41.3)		
Age, yrs (mean ± SD)	63.9 ± 8.4	64.5 ± 8.1	63.2 ± 8.6	1.013∗	0.312
BSA	1.83 ± 0.14	1.84 ± 0.14	1.82 ± 0.15	1.033∗	0.303
BMI, *n* (%)					
≥25	109 (60.9)	62 (71.3)	47 (51.1)	7.645^#^	0.006
<25	70 (39.1)	25 (28.7)	45 (48.9)		
Tobacco use, *n* (%)	54 (30.2)	27 (31.0)	27 (29.3)	0.060^#^	0.806
Alcohol use, *n* (%)	15 (8.4)	7 (8.0)	8 (8.7)	0.025^#^	0.875
Hypertension, *n* (%)	107 (59.8)	55 (63.2)	52 (56.5)	0.834^#^	0.361
Hyperlipidemia, *n* (%)	91 (50.8)	52 (59.8)	39 (42.4)	5.404^#^	0.020
Diabetes mellitus, *n* (%)	35 (19.6)	19 (21.8)	16 (17.4)	0.562^#^	0.453
Coronary disease, *n* (%)	79 (44.1)	40 (46.0)	39 (42.4)	0.233^#^	0.629
AF, *n* (%)					
Prxm AF	93 (52.0)	44 (50.6)	49 (53.3)	0.129^#^	0.719
Pst or pmnt AF	86 (48.0)	43 (49.4)	43 (46.7)		
AF duration (yrs [md(Q1-Q3)])	4 (2-8)	5 (3-9)	4 (2-7)	-2.995∗∗	0.003
CHA_2_DS_2_-VASc score, *n* (%)					
≥2	131 (73.2)	65 (74.7)	66 (71.7)	0.201^#^	0.654
<2	48 (26.8)	22 (25.3)	26 (28.3)		
Anticoagulant use, *n* (%)	19 (10.6)	8 (9.2)	11 (12.0)	0.359^#^	0.549

Numerical data are expressed as the mean ± standard deviation. Categorical data as numbers (percentages). Nonparametric data are expressed as the median (interquartile range). BSA: body surface area; BMI: body mass index; AF: atrial fibrillation; Prxm AF: paroxysmal atrial fibrillation; Pst or pmnt AF: persistent or permanent atrial fibrillation, respectively. ^#^*X*^2^ value, ∗*t* value, ∗∗*Z* value.

**Table 2:** Comparison of left atrial appendage parameters between the two groups.

Characteristics	Total (*n* = 179)	Cases (*n* = 87)	Controls (*n* = 92)	*t* value	*P* value
LAAODmax (cm)	3.14 ± 0.41	3.31 ± 0.38	2.97 ± 0.38	5.862	<0.001
LAAODmax Index (cm/m^2^)	1.72 ± 0.23	1.80 ± 0.21	1.64 ± 0.24	4.783	<0.001
LAAODmin (cm)	2.05 ± 0.35	2.18 ± 0.32	1.93 ± 0.33	5.212	<0.001
LAAODmin Index (cm/m^2^)	1.12 ± 0.19	1.19 ± 0.17	1.06 ± 0.19	4.647	<0.001
LAAODmax/LAAODmin	1.55 ± 0.18	1.53 ± 0.16	1.56 ± 0.21	−1.280	0.202
LAAOA (cm^2^)	5.33 ± 1.37	5.90 ± 1.36	4.80 ± 1.14	5.820	<0.001
LAAOA Index (cm^2^/m^2^)	2.92 ± 0.73	3.20 ± 0.71	2.65 ± 0.64	5.481	<0.001
LAAD (cm)	4.53 ± 0.65	4.61 ± 0.56	4.45 ± 0.71	1.579	0.116
LAAD Index (cm/m^2^)	2.49 ± 0.39	2.51 ± 0.31	2.46 ± 0.44	0.801	0.425
LAAVmax (ml)	13.26 ± 3.67	14.58 ± 3.73	12.02 ± 3.16	4.946	<0.001
LAAVmax Index (ml/m^2^)	7.24 ± 1.91	7.91 ± 1.92	6.61 ± 1.68	4.826	<0.001
LAAVmin (ml)	7.93 ± 2.84	9.27 ± 2.69	6.66 ± 2.38	6.877	<0.001
LAAVmin Index (ml/m^2^)	4.33 ± 1.50	5.03 ± 1.40	3.67 ± 1.28	6.823	<0.001
LAAEF(%)	40.86 ± 11.23	36.20 ± 10.54	45.25 ± 10.07	−5.875	<0.001

LAAODmax and LAAODmin: maximum and minimum left atrial appendage orifice diameter, respectively; LAAODmax/LAAODmin: ratio of LAAODmax to LAAODmin; LAAOA: left atrial appendage orifice area; LAAD: left atrial appendage depth; LAAVmax and LAAVmin: maximum and minimum left atrial appendage volume; one value index: ratio of the one value to body surface area (BSA); LAAEF: left atrial appendage emptying fraction.

The article "Coronary CTA to Investigate Predictive Value of Left Atrial Appendage for Cardiogenic Stroke in Patients with Nonvalvular Atrial Fibrillation" was published in 2020. Journal: Biomed Res Int.

**Table 3:** Binary logistic regression results to identify independent predictors of cardiogenic stroke.

Variable	Odds ratio	95% confidence interval for odds ratio	*P* value
*LAAOA Index (cm* ^2^ */m* ^2^)			
≤ 2.36			0.005
2.37~2.86	1.799	0.693~4.670	0.228
2.87~3.48	1.930	0.726~5.129	0.187
3.49+	5.826	2.167~15.661	<0.001
*LAAEF (%)*			
51.13+			<0.001
41.79~51.12	1.628	0.613~4.321	0.328
30.37~41.78	3.081	1.166~8.139	0.023
≤30.36	8.255	2.929~23.264	<0.001

Abbreviations as in Table 2.

## Data Availability

The testing methods and experimental data used to support the findings of this study are included within the article.
